The article "Optical rectification and absorption coefficients studied by a short-range topless exponential potential well with inverse square root" was retracted in 2020. Reasons: errors in the analysis; unreliable results or conclusions.

# Optical rectification and absorption coefficients studied by a short-range topless exponential potential well with inverse square root

**DOI:** 10.1038/s41598-019-38519-5

**Published:** 2019-02-19

**Authors:** Qiucheng Yu, Kangxian Guo, Meilin Hu

**Affiliations:** 1 Department of Physics, School of Physics and Electronic Engineering, Guangzhou University, Guangzhou, 510006 China; 2 Guangdong Provincial Engineering and Technology Research Center of Semiconductor Lighting and Backlighting, Guangzhou, 510006 China; 3 Dipartimento di Fisica, Universitàdi Napoli Federico II, Complesso universitario di Monte Sant’Angelo, via Cintia, Napoli, 80126 Italy

## Abstract

A topless potential energy with inverse square root is introduced to solve the energy spectrum equations and the bound state wave functions of the static Schrödinger equation by coordinate variation and combining the extraordinary coefficients of the confluent hypergeometric functions. Furthermore, the model of optical rectification (OR) and absorption coefficients (AC) with this special potential energy *V*(*x*) will appear regular changes. In this work, we explore the specific characteristics of the OR and AC with the inverse square root potential through multiple factors such as energy intervals and matrix elements.

## Introduction

The relativistic wave equation has received extensive attentions due to the developments of piecewise continuous potential^1,2^ and the super-symmetric quantum mechanics^3,4^. Also, in recent years, there have been many new researches in integrable^5^ and non-analytical potentials^6^. In this paper, we combine these two issues to introduce a more accurate integrable potential, which is short-range potential energy with inverse exponential root, and it vanishes exponentially at infinity. Such a topless exponential potential well belongs to the Heun potential that first discussed by Lemieux and Bose in 1969^7–9^.

In addition, the researches of the Schrödinger equation of some special models are the basic method for studying complex problems, they are also the eternal hotspot of quantum technology^10–15^. It can be found that the bound states of the Heun potential class is finite^16,17^, that is, the wave functions of bound state which can vanish at infinity and origin. Such special wave functions can have an important effect on nonlinear optical properties^18–20^.

Nonlinear optics is a new field in optical theories which is becoming more and more mature^21–25^. And now it has been done well in experiments^26–28^. The optical rectification effect is a process of generating a low-frequency electrode field (THz) by the interaction of a pulsed laser and a nonlinear medium, and belongs to a special nonlinear optical effect^29,30^. Besides, under the action of strong laser, the absorption coefficients of the mediums will change with the light intensity, which has extensive roles on nonlinear optical theory, material structure, and terahertz technology^31,32^. Here the solution of the topless potential energy formed by the inverse square singularity is brought into OR and AC, and the new effects formed by energy intervals and matrix elements are analyzed in detail.

## Theoretical Framework

### Solution of the Schrödinger equation with exponential potential

In this paper, we introduce an inverse square root potential energy

1 $$V=\frac{{V}_{k}}{\sqrt{z}}=\frac{{V}_{k}}{\sqrt{1-{e}^{-x/a}}}\mathrm{.}$$

Here *z* is defined as a short-range exponential function *z* = 1 − *e*^−*x*/*a*^, and *V*_*k*_ is the variable of the potential. Then the expression of potential energy *V*(*x*) is obtained:

2 $$V(x)=\frac{{V}_{k}}{\sqrt{1-{e}^{-x/a}}}\mathrm{.}$$

The potential well *V*(*x*) defined on the positive half axis (blue line) is plotted in Fig. 1, as well as its two asymptotic fitting curves. $V{|}_{x\to 0}={V}_{k}+\frac{{V}_{k}}{\sqrt{x/a}}$ is the exponential asymptote of *z* → 0 (green line), and $V{|}_{x\to +\infty }={V}_{k}+\frac{{V}_{k}{e}^{-x/a}}{2}$ is the asymptote of *x* → +∞ (brown line). Figure 2 are three-dimensional representations of potential energy *V*(*x*). From this, we can clearly see that it is a short-range potential energy without top.

**Figure 1:** Transformation of coordinates *x* and *z*. Inverse square root topless exponential potential *V*(*x*) and its approximations.

**Figure 2:** Three-dimensional pictures of the topless exponential potential *V* and its projection.

Bring the above potential energy into the one-dimensional fixed Schrödinger equation with mass *m* and energy *E*

3 $$\frac{{d}^{2}\varphi }{d{x}^{2}}+\frac{2m\varphi }{{\hslash }^{2}}(E-V(x))=0,$$

the Heun equation can be gotten by transforming the independent variables *z* = *z*(*x*) = 1 − *e*^−*x*/*a*^ and dependent variables *ϕ* = *u*(*z*)*ψ*(*z*):

4 $${u}_{zz}+(\frac{2{\psi }_{z}}{\psi }+\frac{{\sigma }_{z}}{\sigma }){u}_{z}+(\frac{{\psi }_{zz}}{\psi }+\frac{{\psi }_{z}{\sigma }_{z}}{\psi \sigma }+\frac{2m\,(E-V(z))}{{\sigma }^{2}\hslash })\,u=0,$$

where

5 $$\sigma =\frac{dz}{dx}=\frac{\mathrm{(1}+z\mathrm{)(1}-z)}{2az}.$$

We expand the solution of the Heun equation *u* into a Taylor series $u=\sum _{n=0}^{\infty }\,{c}_{n}{z}^{n}$, where *c*_0_ ≠ 0. After continuously calculating the coefficient *c*_*n*_, the hypergeometric representation of the Taylor series solution is found. The hypergeometric reduction is achieved by a common single-item transformation involving confluent hypergeometric function _1_*F*_1_, which can obtain a general solution of Schrödinger equation with topless potential energy:

6 $$\varphi =u({c}_{1}+{c}_{2}){(z+1)}^{{\xi }_{1}}{(z-1)}^{{\xi }_{2}},$$

where

7 $${\xi }_{1}=\pm \sqrt{\frac{2m{a}^{2}}{{\hslash }^{2}}(2{V}_{k}-E)},\,{\xi }_{2}=\mp \,\sqrt{\frac{2m{a}^{2}E}{{\hslash }^{2}}}.$$

And *u* is defined as:

8 $$u=({c}_{1}\ast {}_{1}F_{1}(-\frac{\gamma }{2};\frac{1}{2};{y}^{2})+{c}_{2}H(y)){e}^{-y\sqrt{2\gamma }}.$$

Here _1_*F*_1_ is the hypergeometric function, the auxiliary dimensionless parameter *y* represents coordinate scaling after deformation that $y=\sqrt{2\gamma }+\sqrt{\beta z}\ast {\rm{sgn}}\,({V}_{k})$, *c*_1_, *c*_2_ are arbitrary constants and *H* is a Hermite function. The relevant parameters are:

9 $$\beta =\sqrt{\frac{-8mE}{{\hslash }^{2}}},\,\gamma =\frac{{m}^{2}{V}_{k}^{2}}{{(-2mE)}^{\frac{3}{2}}\hslash }.$$

Let *γ* = *n* and *n* ∈ *N*, we can derive the bounded quasi-polynomial solution of the standard set of energy levels, that is, *u* (Eq. (8)) can be written as a Hermite polynomial. In order to ensure that the solution of potential energy disappears at infinity, taking *c*_1_ = 0, then the general expression of the energy levels can be educed:

10 $${E}_{n}={(\frac{-m{V}_{k}}{{\hslash }^{2}})}^{\frac{1}{3}}\frac{{V}_{k}}{2}\ast {n}^{-2/3},\,n=1,2,3,\ldots .$$

Figure 3 is a schematic diagram of the energy levels in which the energy interval *E*_21_ = *E*_2_ − *E*_1_ increases with the growth of *V*_*k*_. The increase of *E*_21_ also indicates the increment of *ω*_21_ with ${\omega }_{ij}=\frac{{E}_{j}-{E}_{i}}{hbar}$, which represents that the peak value of nonlinear optical characteristics will augment as the potential coefficient *V*_*k*_ increases. And the corresponding wave functions are as follows:

11 $${\varphi }_{n}=({H}_{n}(y)-\sqrt{2n}{H}_{n-1}(y)){e}^{-\sqrt{2n}y-\beta x/2},$$

where $y=\sqrt{2n}+\sqrt{\beta x}$. We list the first four terms of Eq. (11) for ease of calculation, which is presented in the upper right corner of Fig. 4.

12 $${\varphi }_{1}=(\,-\,\sqrt{2}y+1){e}^{-\frac{\beta }{2}x-\sqrt{2}y},$$

13 $${\varphi }_{2}=\mathrm{(3}{y}^{2}-3y-\mathrm{2)}{e}^{-\frac{\beta }{2}x-2y},$$

14 $${\varphi }_{3}=(\,-\,2\sqrt{6}{y}^{3}+6{y}^{2}+3\sqrt{6}y-3){e}^{-\frac{\beta }{2}x-\sqrt{6}y},$$

15 $${\varphi }_{4}=(3\sqrt{4}{y}^{4}-4\sqrt{6}{y}^{3}-5\sqrt{8}{y}^{2}+15y+4){e}^{-\frac{\beta }{2}x-\sqrt{8}y}.$$

**Figure 3:** Relationship between energy interval *E*_21_ and potential parameter *V*_*k*_.

**Figure 4:** First four terms of the wave functions *ϕ*_*x*_.

As can be seen from the figure, each wave function has a different assignment at the origin. When discussing the case where the bound-state wave functions vanish at infinity and the origin, we should normalize the energy levels and derive an exact approximation of the energy spectrum:

16 $${E}_{n}={(\frac{-m{V}_{k}}{{\hslash }^{2}})}^{\frac{1}{3}}\frac{{V}_{1}}{2}{(n-\frac{1}{2\pi })}^{-2/3},\,n=1,2,3,\ldots .$$

In this way, the wave functions can be influenced by the change of the coefficient *γ* (Eq. (9)) in order to obtain the bound-state wave functions. This is indeed a fairly accurate approximation which is also made in Fig. 4. For all *n* > 2, the relative error is less than 10^−3^. For *n* ≥ 7, the relative error is less than 10^−5^.

### The optical rectification and absorption coefficients

First of all, it is well known that the Liouville equation with density matrix operator is an important formula for discussing nonlinear optics

17 $$\frac{\partial {\rho }_{ij}}{\partial t}=\frac{1}{i\hslash }{[{H}_{0}-ME(t),\rho ]}_{ij}+{{\rm{\Gamma }}}_{ij}{({\rho }^{(0)}-\rho )}_{ij},$$

where *M* is the matrix element, *H*_0_ represents the zero-order Hamiltonian with no optical field effect, Γ_*ij*_ indicates the relaxation rate that Γ_*ij*_ = 1/*T*_0_ = Γ_0_ (*i* ≠ *j*). And *E*(*t*) in Eq. (17) reveals the electric field of light that its expression is

18 $$E(t)={E}_{0}\,\cos \,(\omega t)=\tilde{E}\,\exp \,(i\omega t)+\tilde{E}\,\exp \,(\,-\,i\omega t),$$

which can be expressed by means of electric polarization

19 $$\begin{array}{rcl}P(t) & = & {\varepsilon }_{0}{\chi }_{\omega }^{(1)}\tilde{E}{e}^{i\omega t}+{\varepsilon }_{0}{\chi }_{0}^{(2)}{\tilde{E}}^{2}+{\varepsilon }_{0}{\chi }_{2\omega }^{(2)}{\tilde{E}}^{2}{e}^{2i\omega t}\\  &  & +{\varepsilon }_{0}{\chi }_{3\omega }^{(3)}{\tilde{E}}^{3}{e}^{3i\omega t}+{\varepsilon }_{0}{\chi }_{\omega }^{(3)}{\tilde{E}}^{3}\tilde{E}{e}^{i\omega t}+{c}{.c}{.}\end{array}$$

The five parameters ${\chi }_{\omega }^{\mathrm{(1)}}$, ${\chi }_{0}^{\mathrm{(2)}}$, ${\chi }_{2\omega }^{\mathrm{(2)}}$, ${\chi }_{3\omega }^{\mathrm{(3)}}$, ${\chi }_{\omega }^{\mathrm{(3)}}$ above are separately the linear polarization, optical rectification coefficients, the second-harmonic coefficients, the third-harmonic coefficients and the third-order polarizability. $\tilde{E}$ represents the half-amplitude of electric field and *c*.*c* in Eq. (18) indicates its complex conjugation.

The iterative method is a practical method for dealing with nonlinear optical coefficients

20 $$\rho (t)=\sum _{n}{\rho }^{(n)}\,(t),$$

and it allows the polarization strength to be expressed as

21 $$P(t)=\frac{1}{V}Tr(\rho M),$$

whose multilevel expression is

22 $${P}^{(n)}(t)=\frac{1}{V}Tr({\rho }^{(n)}M\mathrm{).}$$

Similarly, the Liouville equation can be expressed in the following form:

23 $$\frac{\partial {\rho }_{ij}^{(n+1)}}{\partial t}=\frac{1}{i\hslash }\{{[{H}_{0},{\rho }^{(n+1)}]}_{ij}-i\hslash {{\rm{\Gamma }}}_{ij}{\rho }_{ij}^{(n+1)}\}-\frac{1}{i\hslash }{[M,{\rho }^{(n)}]}_{ij}E(t).$$

By bringing the different expressions of Eq. (22) into the Liouville equation Eq. (23), the different coefficients of nonlinear optics can be obtained. Firstly, the expression of the linear polarizability is

24 $${\chi }_{0}^{(2)}={M}_{12}^{2}{\delta }_{12}\frac{4e{\sigma }_{\upsilon }}{{\varepsilon }_{0}{\hslash }^{2}}\frac{{\omega }_{12}^{2}(1+{{\rm{\Gamma }}}_{2}/{{\rm{\Gamma }}}_{1})+({\omega }^{2}+{{\rm{\Gamma }}}_{2}^{2})({{\rm{\Gamma }}}_{2}/{{\rm{\Gamma }}}_{1}-1)}{[{({\omega }_{12}-\omega )}^{2}+{{\rm{\Gamma }}}_{2}^{2}][{({\omega }_{12}+\omega )}^{2}+{{\rm{\Gamma }}}_{2}^{2}]}.$$

Then the coefficient of the optical rectifications is as follows

25 $${\chi }^{(1)}(\omega )=\frac{{|{M}_{ij}|}^{2}}{{\varepsilon }_{0}(\hslash \omega -\hslash {\omega }_{ij}+i\hslash {{\rm{\Gamma }}}_{ij})}.$$

Finally, form the of third-order nonlinear polarizability is given by

26 $${\chi }_{\omega }^{(3)}=\frac{{e}^{4}{\sigma }_{\upsilon }}{{\varepsilon }_{0}{\hslash }^{3}}\frac{|{M}_{12}{M}_{23}{M}_{34}{M}_{41}|}{(\omega -{\omega }_{21}+i{{\rm{\Gamma }}}_{21})(2\omega -{\omega }_{31}+i{{\rm{\Gamma }}}_{31})(3\omega -{\omega }_{41}+i{{\rm{\Gamma }}}_{41})}.$$

${M}_{ij}= < \,i|M|j >$ above reveals the matrix elements of dipole transition, and *σ*_*υ*_ is the difference of electron density with ${\sigma }_{\upsilon }=\frac{{\rho }_{jj}^{\mathrm{(0)}}-{\rho }_{ii}^{\mathrm{(0)}}}{V}$.

Regarding the nonlinear optical absorption coefficients, it is known that the relationship between the real part and the imaginary part of the polarization rate is that

27 $$\alpha (\omega )=\omega \sqrt{\frac{\mu }{{\varepsilon }_{R}}}\,{Im}\,({\varepsilon }_{0}\chi (\omega )).$$

Here, *μ* is the permeability of the system, *ε*_*R*_ is the real part of the dielectric constant (${\varepsilon }_{R}={n}_{r}^{2}$), and *n*_*r*_ represents the refractive index of the medium. Put ${\chi }_{\omega }^{\mathrm{(1)}}$ (Eq. (25)) into the formula above (Eq. (27)), the linear-optical absorption coefficient can be obtained

28 $${\alpha }^{(1)}(\omega )=\omega \sqrt{\frac{\mu }{{\varepsilon }_{R}}}\frac{|{M}_{21}{|}^{2}{\sigma }_{\upsilon }\hslash {{\rm{\Gamma }}}_{0}}{{({E}_{21}-\hslash \omega )}^{2}+{(\hslash {{\rm{\Gamma }}}_{0})}^{2}}.$$

Similarly, the nonlinear-optical absorption coefficients can be gotten after putting ${\chi }_{\omega }^{\mathrm{(3)}}|\tilde{E}{|}^{2}$ into Eq. (27)

29 $$\begin{array}{rcl}{\alpha }^{(3)}(\omega ,I) & = & -\omega \sqrt{\frac{\mu }{{\varepsilon }_{R}}}(\frac{I}{2{\varepsilon }_{0}{n}_{r}c})\frac{|{M}_{21}^{2}{|}^{2}{\sigma }_{\upsilon }\hslash {{\rm{\Gamma }}}_{0}}{{[{({E}_{21}-\hslash \omega )}^{2}+{(\hslash {{\rm{\Gamma }}}_{0})}^{2}]}^{2}}\\  &  & \,\times \,\{4|{M}_{21}{|}^{2}-\frac{|{M}_{22}-{M}_{11}{|}^{2}[3{E}_{21}^{2}-4{E}_{21}\hslash \omega +{\hslash }^{2}({\omega }^{2}-{{\rm{\Gamma }}}_{0}^{2})]}{{E}_{21}^{2}+{(\hslash {{\rm{\Gamma }}}_{0})}^{2}}\}.\end{array}$$

Hence the total optical absorption coefficients can be written as

30 $$\alpha (\omega ,I)={\alpha }^{(1)}(\omega )+{\alpha }^{(3)}(\omega ,I),$$

where *I* is the light intensity of the incident light with $I=2{\varepsilon }_{0}{n}_{r}c{\tilde{E}}^{2}$.

## Results and Discussions

The section here is mainly be used to study the special phenomenons of optical rectification and optical absorption coefficients under the action of this special potential energy. And the parameters to be used in this part are ${m}_{0}^{\ast }=0.067\,{m}_{0}({m}_{0}=9.10956\times {10}^{-31}\,kg)$, *ε*_0_ = 8.85 × 10^−12^, *μ* = 4*π* × 10^−7^ *Hm*^−1^, *T*_0_ = 0.14 *ps*, Γ_*ij*_ = 1/(0.14 × 10^−12^)*s*^−1^, and *σ*_*υ*_ = 5.0 × 10^22^ *m*^−3^.

### The optical rectification

Figure 5 mainly shows the comparison of the optical rectification coefficient under the influence of exponential potential well *V* (*V*_*k*_ = 20 *nm*) and the normal case. It can be seen from the figure that the short-range exponential potential can make the intensity of optical rectification become larger and cause blue-shift phenomenon. As a whole, the reason is that such a special exponential potential energy can adjust the matrix elements of the function *M*_*ij*_ to a higher level, and the increment of matrix elements will make the intensity and peak value of the optical rectification become larger.

**Figure 5:** Comparison of optical rectification in classical potential and exponential potential.

The curves of the product of matrix product ${M}_{21}^{2}{\delta }_{21}$ and its individual elements *M*_21_, *δ*_21_ (*δ*_21_ = |*M*_22_ − *M*_11_|) are plotted in Fig. 6, which reveals that the decrease of the absolute value of *M*_21_ basically set a tone of the trend of the matrix-element product that OR reduces with the increase of *V*_*k*_. This also shows that the peak value of the optical rectification in this case will become smaller.

**Figure 6:** The graphs of matrix elements and their product with the change of *V*_*k*_.

Figure 7 can better illustrate the feature of Fig. 6 above. We take the graph of OR coefficients ${\chi }_{0}^{\mathrm{(2)}}$ with different values of *V*_*k*_ and put them together in Fig. 7. It can be found that as the potential coefficient *V*_*k*_ increases, the intensity of the optical rectification is weakened. The fitting curve of the highest points are also showing the trend of the matrix-element product ${M}_{21}^{2}\ast {\delta }_{21}$ in Fig. 6. Another phenomenon is that with the increment of *V*_*k*_, the optical rectification tends to be larger incident photon energy *ħω*, that is, the blue shift phenomenon occurs, which is due to the growth of the energy interval *E*_21_ in Fig. 3. With the augment of *V*_*k*_, the energy interval that monotonically increasing demonstrates ${\chi }_{0}^{\mathrm{(2)}}$ in this case have larger energy regions.

**Figure 7:** Global presentation of optical-rectification coefficients with multiple *V*_*k*_.

### The absorption coefficients

The three optical absorption coefficients (linear-optical absorption coefficient *α*^(1)^, nonlinear-optical absorption coefficient *α*^(3)^ and total optical absorption coefficients *α*) with or without potential energy *V* are displayed together in Fig. 8 when *V*_*k*_ = 30 *nm* and *I* = 3 × 10^9^ *W*/*m*^2^. It can be seen that under the influence of such topless potential, the intensity of the linear-optical absorption coefficient is increased, and conversely, the absorption coefficient of the nonlinear optical is reduced. This is also because the exponential potential *V* will make the matrix element *M* have a significant enhancement compared with the general case without *V*. And as can be seen from Eq. (28) and Eq. (29), the increased *M*_21_ can cause *α*^(1)^ to increase and *α*^(3)^ to decrease. The OA coefficient under the influence of *V* will also appear in the larger incident-photon energy region *ħω* due to the raise of *E*_21_.

**Figure 8:** Comparison of optical-absorption coefficients in inverse square root exponential potential well and original one-dimensional infinite well.

In Fig. 9, we plot the curves of matrix elements *M*_21_, *M*_22_ − *M*_11_ and their squares in equations of linear-optical absorption coefficient *α*^(1)^ (Eq. (28)) and the nonlinear-optical absorption coefficient *α*^(3)^ (Eq. (29)). As *V*_*k*_ becomes larger, all of the matrix elements increase semi-exponentially. While (*M*_22_ − *M*_11_)^2^ has the largest value-added, which indicates the growths about *α*^(1)^ and *α*^(3)^.

**Figure 9:** Different forms of matrix elements as a function of *V*_*k*_.

Figure 10 below shows seven optical-absorption coefficients by a method of collectively presenting multiple parameters *V*_*k*_, whose trend satisfies the enhancement in the strength of *α*^(1)^ and *α*^(3)^ that mentioned above. The total optical-absorption coefficient also shows an increasing trend due to the large increase of *α*^(1)^. Similarly, we use the orange curve to connect the vertices of *α*^(1)^ and *α*^(3)^, and what can be seen is that the growth trend of their intensities are a semi-exponential type consistent with the matrix elements.

**Figure 10:** Global presentation of optical-absorption coefficients with multiple variable *V*_*k*_.

We know that the intensity of light has a great influence on the absorption coefficient, as well as the change of the *α* in the Fig. 11: the greater intensity of the light causes multiple peaks in the total light absorption coefficient *α*, producing an oscillating effect. The smaller light intensity will make the optical-absorption coefficient produce bleaching, and only appear a regular apex. In this paper, the total OA coefficient *α* is divided into linear one *α*^(1)^ and nonlinear one *α*^(3)^, and the conditions under different illumination are shown together in Fig. 11. As can be observed, the curve of linear optical-absorption coefficient does not change with the change of light intensity (blue lines), while the nonlinear OA coefficient enhances with the augment of light intensity, and the peak value increases in the opposite direction. From Eq. (29), we can also see that the light intensity *I* has an important influence on *α*^(3)^.

**Figure 11:** Different manifestations of three optical-absorption coefficients under different light intensities.

## Conclusion

The short-range topless potential energy that exhibits as an inverse exponential root at the origin and vanishes exponentially at the infinity, is studied in this paper. By using the confluent hypergeometric function, we can obtain the exact spectral equations and the solution of wave functions. The energy interval *E*_21_, which becomes larger as *V*_*k*_ increases, indicates that the optical rectification and optical-absorption coefficients tend to a larger incident photon energys *ħω* as the *V*_*k*_ increases, that is, a blue shift occurs. And the trend of matrix elements with *V*_*k*_ is also the tendency of peak value of OR and AC.

The paper is an exploration of the specific characteristics of nonlinear optics with a special model. It is hoped that our paper will bring new enlightenment and research power to readers. Furthermore, we holp it will have a certain influence on the research process of nonlinear optics and can promote the development of low-dimensional systems.
